# Research on Management Efficiency and Dynamic Relationship in Intelligent Management of Tourism Engineering Based on Industry 4.0

**DOI:** 10.1155/2022/5831062

**Published:** 2022-01-22

**Authors:** Tianchen Hou

**Affiliations:** Physical Education College of Zhengzhou University, Zhengzhou 450044, Henan, China

## Abstract

The digital age of artificial intelligence marks the rapid development of tourism engineering and the gradual improvement of intelligent management theory. This study aims to solve the problems of low efficiency of dynamic relationship analysis and low data utilization in traditional intelligent management methods of tourism engineering. This work studies the dynamic optimization model of tourism engineering management theory based on the artificial intelligence data analysis model and designs the dynamic analysis model of tourism engineering management data based on the convolution neural network. The model can collect dynamic data information of tourism management from many aspects and can also be used to study and analyze human behavior patterns based on the convolutional neural network algorithm. According to the human behavior data analysis model and convolution neural network algorithm, this study formulates the real-time management data scheme of tourism engineering and better extracts the characteristic information of the dynamic data of tourism engineering management. The results show that the topology optimization model of tourism intelligent management based on the convolutional neural network achieves high feasibility, high data accuracy, and high response speed. It can improve the collaborative coupling relationship between management efficiency and dynamic data in tourism engineering management based on big data analysis technology. It realizes the effective combination of tourism management, digital management, and artificial intelligence algorithm.

## 1. Introduction

At present, the traditional “many to many” cluster point information collection is the main data information of tourism project management in China [1]. Since the beginning of the 21st century, the rapid development of artificial intelligence technology in China has also led to the transformation of data analysis methods in tourism engineering management in China. The emergence of modern tourism engineering management analysis methods such as intelligent tourism management theory planning, efficient management data analysis, and coordinated utilization of software and hardware has contributed to the large-scale promotion of “intelligent management of industrial 4.0 tourism engineering” and provides opportunities [2]. Therefore, diversification and high efficiency have become important features of the intelligent degree of tourism project management in China [3]. At present, although the existing intelligent management system of tourism engineering provides a large number of data information extraction schemes, it is difficult to select a targeted topological representation scheme according to its management dynamic theoretical system and the law of human behavior in the process of dynamic management, so as to achieve the optimal effect of topological analysis [4]. Based on this, this study proposes a theoretical topology analysis model of intelligent management of tourism engineering in the digital age based on big data and the convolutional neural network algorithm.

Aiming at the problems of low data analysis efficiency, low data storage efficiency, and low data classification efficiency existing in the current theoretical analysis model of intelligent management of tourism engineering, this work studies the data mining model scheme of discrete dynamic analysis based on the convolution neural network algorithm and collaborative processing of big data in the cloud, which is mainly divided into four parts.  Section 1 introduces the research background and the overall framework of this study.  Section 2 introduces the research status of intelligent management theory and application methods of tourism engineering.  Section 3 constructs the theoretical topology model of intelligent management of tourism engineering in the digital age based on big data and convolution neural network algorithm, adopts the multilayer convolution perception neural network factor method, and constructs the evaluation index system of tourism management data analysis and intelligent classification objectives of artificial intelligence analysis. In Section 4, the quantitative effect of data analysis of the industrial 4.0 tourism project intelligent management efficiency dynamic analysis model constructed in this study is experimentally analyzed and verified, and a conclusion is drawn in Section 5.

Compared with the data mining model established by the traditional intelligent management analysis model in tourism engineering, which takes the continuity of static management data as the main research object, the innovation of this study is that the discrete dynamic modeling technology and big data topology analysis strategy based on the convolution neural network algorithm are applied to the dynamic analysis model of industry 4.0 tourism engineering management. It can make full use of a large number of dynamic management data, extract appropriate management data feature information, realize the integrity approach at the simulation level, and quantitatively describe the quantitative representative eigenvalues, similarity of multidimensional management analysis modes, and expected evaluation indicators of different tourism projects in the process of employee management scheme allocation with multitransformed neural network factors. It can efficiently carry out customized analysis on the factors affecting management efficiency and accuracy.

## 2. Related Work

Although the domestic management theory analysis model has been developed for several years, there are still some deficiencies in the establishment, operation, and upgrading of the sports data mining model compared with some more developed countries [5]. Wei et al. optimized the data analysis process according to the management principle of three-dimensional space. His team proposed that attention should be paid to the development of the three-dimensional basic structure or dynamic theoretical decomposition method of tourism management based on Gaussian mixture [6]. Masterson et al. proved through experiments that the classified data analysis method can play a good role in differential learning, effectively improve the mining efficiency of big data, and use a number of indicators to evaluate the data analysis ability of the tourism management dynamic analysis model [7]. Greatbatch et al. have verified through repeated practice. The final results show that the establishment method based on human behavior discrete modeling technology can improve the data analysis efficiency of the data mining model and the effectiveness of modifying data. It is suitable for the outside world to carry out continuous R&D planning for tourism engineering management data and find the optimal data structure scheme [8]. Mayro et al. put forward a new group tourism project management data model and database establishment method based on industry 4.0. The multidimensional spatial framework sequence is used to redistribute the data packets of each layer of the original management database, so as to realize the optimal determination of various mining methods in the process of management data capture [9]. According to the traditional establishment mode and practical experience of the data collection system in a general sense, Lang et al. found that the current data mining model has the problems of difficult dimension calculation and poor physical quantity in the process of managing tourism dynamic data analysis. Therefore, they developed a new intelligent data analysis technology based on deep learning [10]. Through logical analysis, adjustment, and summary of different data mining models, Egevad et al. finally established a new data mining system, which can realize delayed capture and real-time feedback of tourism engineering management data [11]. Scholars from Safarnejad L and other universities put forward a new data mining model establishment method based on the multirelationship recommendation algorithm according to the multifactor relationship theory in philology, analyzed the correlation of different modules in the traditional data mining model, and established a double factor analysis model [12]. Verganti et al. comprehensively evaluated the employee management data mining model of a tourism project from the aspects of the selection of the structure form of the tourism management storage database, the classification of the content, and the storage capacity of the database and realized the simulation of the working process of the model database by capturing different types of data [13]. The research results of Kai et al. show that the “data outside” interaction model based on discrete dynamic modeling technology is better than the traditional interaction model in terms of motion data information acquisition ability [14]. In order to improve the acquisition efficiency of tourism engineering management data and the maximum utilization of storage space, Liu et al. conducted various research studies and analyses on different tourism engineering management data and finally classified different data types into various types of data models to avoid storing duplicate data and increase the collection efficiency of tourism data [15]. Goodarzian et al. proved through experiments that the discrete data mining model established can realize the static segmentation of dynamic data and solve the problem that it is difficult to obtain dynamic data in management, but there is a problem of small application range [16].

To sum up, it can be seen that the current tourism engineering focuses on the data mining management analysis model with the continuity of static management data as the main research object in the establishment of the intelligent management analysis model, but there are some problems in this kind of model research, such as low intelligence and low data utilization [17–19]. On the other hand, although China has done more theoretical analyses and research on the establishment method of the intelligent management and intelligent analysis system of tourism engineering, there is room for progress in the achievement transformation at the actual control level, and there is no establishment of the intelligent multimedia control system model [20, 21].

## 3. Methodology

The development of big data and artificial intelligence in the digital age has brought great opportunities for the digital development of intelligent management of tourism engineering [22]. The most typical algorithm in artificial intelligence technology based on big data idea is the convolution neural network algorithm [23]. The typical convolutional neural network structure is a feed forward network with three or more layers without feedback and no interconnection structure in the layer. The convolutional neural network is also a basic method for self-learning and updating at the data level. The first and last layers are called the input layer and output layer, respectively, and the middle layers are the hidden layer (also known as the middle layer) [24]. In the convolution neural network, the neurons in each layer are fully connected, and there is no connection between the neurons in each layer. The neural network algorithm used in the topological representation of management is an intelligent algorithm with “human biological characteristics” based on the overall structure of human neurons and the direct two-way regulation and automatic processing of neurons by the brain [25]. The data processing process of the convolution neural network algorithm is shown in Figure 1.

When the industrial 4.0 tourism engineering intelligent management data information is processed randomly, the mutual coupling analysis of two-way management information classification and the vector processing analysis of multiple coupling combinations are carried out through a single neuron structure with multiple neuron structure (synapse) characteristics, the management type with high modular demand is found from the total object to be processed, and the probability of being selected for secondary or multiple analysis is high. On the contrary, the probability of objects with low significance of management features being selected for secondary or multiple reusable framework processing is very low. The new generation of tourism project objectives has dynamic characteristics, which need to be compared and analyzed for many times to produce unified management. In this way, after several two-way information interaction cycles, mixed characteristic individuals conforming to the characteristics of artificial intelligence are finally generated, that is, modular unified processing for a certain type of tourism management data local optimization and feature extraction.

### 3.1. Establishment Process of the Multiple Grey Convolution Neural Network Model Based on Data Mining

By checking many factors of multimanagement data, we can judge whether there are closely related factors in various data of intelligent management type of tourism engineering. Tourism information management is a process in which information personnel plan, organize, command, coordinate, and control the tourism information source utilizing information technology. From a microperspective, it includes the management of tourism information content. Macroscopically speaking, it includes the management of tourism information institutions and tourism information systems. In this way, we can not only use the comprehensive average index of these closely related factors or one of them to represent a variety of such factors. In addition, the information carried by these multidata to be processed cannot be seriously distorted. The data analysis process of the convolution neural network topology analysis model based on big data and artificial intelligence strategy is shown in Figure 2.

First, assume that there are *n* data objects to be processed (tourism engineering management information), which are called implementation objects, and each observation object has *m* characteristic data (management characteristic information); the sequence can be obtained as follows:

(1) $$\begin{array}{c} X_{1}=\left(x_{1}\left(1\right),x_{1}\left(2\right),\ldots ,x_{1}\left(n\right)\right),\\ X_{2}=\left(x_{2}\left(1\right),x_{2}\left(2\right),\ldots ,x_{2}\left(n\right)\right),\\ X_{3}=\left(x_{3}\left(1\right),x_{3}\left(2\right),\ldots ,x_{3}\left(n\right)\right),\\ X_{m}=\left(x_{m}\left(1\right),x_{m}\left(2\right),\ldots ,x_{m}\left(n\right)\right). \end{array}$$

Then, calculate the absolute correlation *ε*_*ij*_ between *X*_*i*_ and *X*_*j*_ for all *i* ≤ *j*, *i*, *j*=1,2, ⋯, *m*, and the calculation formula is

(2) $$\begin{array}{c} \varepsilon =1-\sqrt{\frac{X_{m}+X_{m+1}}{X_{m}-X_{m-1}}}. \end{array}$$

The corresponding coding function is obtained according to the correlation degree

(3) $$\begin{array}{c} W\left(x\right)=\frac{7x^{2}+x^{4}+1}{7x^{2}+8x^{3}+5x^{4}+2}\varepsilon_{ii}, \end{array}$$

where *ε*_*ii*_=1; *i*=1,2, ⋯, *m* AA. In this process, the following results can be obtained from the simulation analysis of data types in different dimensions. The simulation results without big data coupling factors for different tourism projects are shown in Figure 3.

The simulation results of dynamic coupling quantity under level 1 big data coupling factor for intelligent management types of different tourism projects are shown in Figure 4.

The simulation results of the two-level big data coupling factor in dynamic characterization of intelligent management types of different tourism projects are shown in Figure 5.

For the intelligent management types of different industrial 4.0 tourism projects, the simulation results of three-level big data coupling factors in dynamic characterization are shown in Figure 5.

It can be seen from Figures 3–6 that the comprehensive utilization rate of the information of the corresponding management database changes with the change of the number of topology analyses when performing different degrees of association calculation and processing (level 0/1/2/3 big data coupling factor) for different data under the dynamic relationship topology model of the convolution neural network algorithm and when the level 3 big data coupling factor is added. There are more and more stable branches of its corresponding topological dynamic structure, and its stability utilization rate is also better and better. This is because in the calculation process, through the computer database information and the preset linear judgment program, some data information can be deeply mined and analyzed, so as to realize the quadratic linear processing of the data after the initial linear analysis. After quadratic linear processing, its stability and data utilization are improved. In this study, the values of the analysis indexes of *n* data objects to be processed are divided into the class grey group, which is called *j* index subclass. The convolution network function of *j* index *k* subclass is recorded as *H*_*j*_^*k*^(*x*).

(4) $$\begin{array}{c} H_{j}^{k}\left(x\right)=\frac{x+x_{j}^{k}\left(1\right)}{x_{j}^{k}\left(2\right)-x_{j}^{k}\left(1\right)},\;x\in \left[x_{j}^{k}\left(1\right),x_{j}^{k}\left(2\right)\right]. \end{array}$$

Among them, *x*_*j*_^*k*^(1) and *x*_*j*_^*k*^(2) are the network nodes, and *x* is the data type.

If the function *H*_*j*_^*k*^(*x*) does not have the first and second turning points *x*_*j*_^*k*^(1) and *x*_*j*_^*k*^(2), *H*_*j*_^*k*^(*x*) is called the lower bound measure convolution network function, which is recorded as *H*_*j*_^*k*^[−, −, *x*_*j*_^*k*^(3), *x*_*j*_^*k*^(4)]. In this system, the corresponding lower bound measure function *f*_*j*_^*k*^(*x*) is

(5) $$\begin{array}{c} f_{j}^{k}\left(x\right)=\frac{x_{j}^{k}\left(4\right)-x}{x_{j}^{k}\left(4\right)-x_{j}^{k}\left(3\right)},\;x\in \left[x_{j}^{k}\left(3\right),x_{j}^{k}\left(4\right)\right]. \end{array}$$

The moderate measure function corresponding to this model is shown in formula (6), and the expression of the whitening weight function of the upper bound measure is formula (7).

(6) $$\begin{array}{c} Q_{j}^{k}\left(x\right)=f_{j}^{k}\left(x\right)=\frac{x_{j}^{k}\left(4\right)-x}{x_{j}^{k}\left(4\right)-x_{j}^{k}\left(2\right)},\;x\in \left[x_{j}^{k}\left(2\right),x_{j}^{k}\left(4\right)\right]. \end{array}$$

(7) $$\begin{array}{c} W_{j}^{k}\left(x\right)=f_{j}^{k}\left(x\right)=\frac{x-x_{j}^{k}\left(1\right)}{x_{j}^{k}\left(2\right)-x_{j}^{k}\left(1\right)}\text{,}\;x\in \left[x_{j}^{k}\left(1\right),x_{j}^{k}\left(2\right)\right]\text{.} \end{array}$$

Among them, *x*_*j*_^*k*^(1), *x*_*j*_^*k*^(2), and *x*_*j*_^*k*^(4) are the network nodes, and *x* is the data type.

### 3.2. Tourism Management Efficiency Based on the Convolutional Neural Network Gaussian Mixture Sparse Representation Data Processing Process of the Dynamic Optimization Model

In this model, in order to better determine the specific significance of management data judgment index in the process of grey linear analysis, carry out factor analysis and provide basis for system decision-making. It is necessary to solve the problem of how to find correlation and measure from random time series. By determining the convolution variable weight linear coefficient, the accuracy of management data mining can be better improved. Therefore, the weighted linear coefficient *σ*_*i*_^*k*^ can be expressed as

(8) $$\begin{array}{c} \sigma_{i}^{k}=\sum_{j=1}^{m}f_{j}^{k}\left(x_{ij}\right)\cdot \eta_{j}^{k},\\ \sigma_{i}=\left(\sigma_{i}^{1},\sigma_{i}^{2},\ldots ,\sigma_{i}^{s}\right)=\left(\sum_{j=1}^{m}f_{j}^{1}\left(x_{ij}\right)\cdot \eta_{j}^{1},\sum_{j=1}^{m}f_{j}^{2}\left(x_{ij}\right)\cdot \eta_{j}^{2},\ldots ,\sum_{j=1}^{m}f_{j}^{s}\left(x_{ij}\right)\cdot \eta_{j}^{s}\right). \end{array}$$

The above formula is called the linear coefficient of the multilayer convolution neural network, and its corresponding linear coefficient matrix is

(9) $$\begin{array}{c} \Sigma =\left(\sigma_{i}^{k}\right)=\left[\begin{array}{cccc} \sigma_{1}^{1} & \sigma_{1}^{2} & \cdots & \sigma_{1}^{s}\\ \sigma_{2}^{1} & \sigma_{2}^{2} & \cdots & \sigma_{2}^{s}\\ \cdots & \cdots & \cdots & \cdots \\ \sigma_{n}^{1} & \sigma_{n}^{2} & \cdots & \sigma_{n}^{s} \end{array}\right]. \end{array}$$

In order to realize data mining of the convolutional neural network linear analysis process, the information of target data needs to be translated into language information that can be recognized by computer through a certain pattern. Therefore, after the feature sparse representation process of the Gaussian mixture industrial 4.0 tourism engineering intelligent management data of the management data, the simulation analysis results of the calculation efficiency of three different types of tourism engineering management data combined with human behavior are shown in Figure 7.

As shown in Figure 7, with the increase of the number of topologies, the stability and computational efficiency of the corresponding tourism engineering intelligent management database are also changing. Because some low-frequency or meaningless management data information is intentionally deleted or deleted, the process is stored through a specific mode. To facilitate the data recovery required by posterror processing operations, form a special data information record and realize the conversion from data information to computer storage information, and its storage function can be expressed as *T*(*x*).

(10) $$\begin{array}{c} T\left(x\right)=\frac{\sum_{j=1}^{m}f_{j}^{1}\left(x_{j}\right)}{\eta_{j}^{1}}. \end{array}$$

Among them, *η*_*j*_^1^ is the storage coefficient, and its sparse representation can be expressed as *T*′(*x*), which can be expressed as

(11) $$\begin{array}{c} T^{\prime }\left(x\right)=\frac{\sum_{j=1}^{m}f_{j}^{1}\left(x_{j}\right)}{\eta_{j}^{1}H\left(x\right)}. \end{array}$$

where *η*_*j*_^1^ is the storage coefficient and *H*(*x*) is the discriminant function.

Choosing different grey linear methods will make the data in the cluster have different correlation degrees. The topology analysis model based on the convolutional neural network is to fuzzy search and screen the unknown data targets (newly collected industry 4.0 tourism project management information and known human behavior data) through data mining of multitarget data. The screening function is *P*(*x*), and the expression is

(12) $$\begin{array}{c} P\left(x\right)=\frac{\sum_{j=1}^{m}\left(x_{j}-\bar{x}\right)}{\eta_{j}^{1}\bar{x}}, \end{array}$$

where *η*_*j*_^1^ is the storage coefficient.

When it is necessary to classify different types of data indicators (such as relevant assessment data indicators of a tourism project), the evaluation model *Z*(*x*) can be expressed as

(13) $$\begin{array}{c} Z\left(x\right)=\frac{1}{\eta_{j}^{1}\sum_{j=1}^{m}\left(x_{j}-\bar{x}\right)}, \end{array}$$

where *η*_*j*_^1^ is the storage coefficient and $\bar{x}$ is the average number of management decomposition information.

(14) $$\begin{array}{c} Z\left(x\right)=\frac{1}{\eta_{j}^{1}\sum_{j=1}^{m}\left(x_{j}-\bar{x}\right)}. \end{array}$$

In the optimal case, the convolution neural network analysis model can realize the recognition of multiple data under a certain similarity. However, there are still some problems in the data mining process and management dynamic algorithm. In order to improve the recognition degree of the association degree between management data information (feature information) and multiple data (management color channel and salient feature) by the multiple grey linear analysis model as much as possible, the expression of the association degree *R*(*x*) is

(15) $$\begin{array}{c} R\left(x\right)=\frac{\eta_{j}^{1}}{\sum_{j=1}^{m}x_{j}-\bar{x}/x_{j+1}+\bar{x}}. \end{array}$$

At present, the most commonly used method is to achieve accurate topological linear analysis through big data database statistics and data comparison between the same management types. The above dynamic flapping analysis method is also used to compare and determine the well-known feature recognition information and management sparse representation pattern information.

## 4. Result Analysis and Discussion

### 4.1. Experimental Design Process and Data Results

The input layer data used in this experiment are the known industry 4.0 tourism engineering management information data, the hidden layer is the artificial intelligence topology analysis strategy based on big data and the convolution neural network algorithm, the output layer is the dynamic optimal selection combination of tourism engineering management, and its convolution learning strategy is the tourism engineering intelligent management rules and regulations and employee level treatment. When evaluating the topological rate and change type of tourism engineering management data, it needs to be evaluated from many aspects. According to the needs of tourism engineering development, this study proposes 25 indicators to evaluate the quality of management topology analysis. Through the observation results of 25 relevant data managing topological-mixed features, the above indicators are properly classified and sparse representation analysis, and the characterization standard is simplified by deleting some unnecessary (i.e., less influential) indicators, so as to realize the quantitative representation of the above data indicators, which is more convincing. During the experiment, the management data of three types (6 groups in total, 2 groups in each type) of different tourism projects are verified by topological analysis. The experimental results are shown in Figure 8.

### 4.2. Analysis of Experimental Results of Management Data Accuracy Based on the Convolutional Neural Network

The analysis results of data accuracy in the experimental results are shown in Figure 9.

From the experimental results shown in Figure 8 and the accuracy analysis results shown in Figure 9, it can be seen that after the analysis of three types of data (two groups each), the corresponding change of topology classification performance index is obvious. Among them, the topology performance of the third group of data is the highest, but the corresponding big data analysis data deviation is also the highest because with the increase of topology structure, the dimension of data analysis is also increasing, so its deviation will also change. On the other hand, among the above data indicators for evaluating the quality of topology analysis, some or several indicators do have correlation or mixed relationships.

In addition, it can be seen from the data shown in Figures 8 and 9 and the experiment that in the process of processing the experimental data, this study adopts an efficient and intelligent topological data analysis method. The model can realize the unified management of sparse representation demand data of different tourism management and different types of management representation method data. According to the local differences between data and the actual needs of sparse representation, the algorithm is used for intelligent optimization, analysis, and processing to realize the high-precision utilization and remote dynamic maintenance of data. Then, through the eigenvalues of the signals collected by the wireless nano data processing equipment and the structural characteristics of different management in the sparse representation process, according to the different eigenvalues such as vector difference and matrix difference, the intelligent optimization processing and deep information mining process based on the machine learning model and neural network algorithm are applied. Realize the classification level division of different management Gaussian mixture feature sparse representation methods in data analysis. Finally, through a series of data analysis processes represented by the neural network algorithm in the sparse representation of tourism management, classify according to the differences of information, realize the high classification of the similarity of different data, and realize the fitting analysis and simulation of approximate or the same data according to the different requirements for the sparse representation of different tourism management. Then, it completes the efficient and high-precision classification of the sparse representation optimization link of managing Gaussian mixture features.

## 5. Conclusion

This work studies the discrete dynamic analysis data mining model scheme based on the convolutional neural network algorithm and big data cloud collaborative processing. Compared with the traditional intelligent management analysis model of tourism engineering, which takes the continuity of static management data as the main research object, the innovation of this study is to apply discrete dynamic modeling technology and big data topology analysis strategy based on the convolution neural network algorithm to the dynamic analysis model of industry 4.0 tourism engineering management. It can make full use of a large number of dynamic management data, extract appropriate management data feature information, realize the simulation level integrity method, quantitatively describe representative quantitative eigenvalues, the similarity of multidimensional management analysis modes and expected evaluation indicators of different tourism projects in the process of employee management scheme allocation, and adopt multiconversion neural network factors. It can efficiently customize and analyze the factors affecting management efficiency and accuracy. However, the algorithm only analyses the impact and correlation degree from the local analysis of management and does not consider other potential factors of sparse representation of management features. Therefore, the comprehensive analysis of the index evaluation system and the influence degree of other factors need to be further studied.

## Figures and Tables

**Figure 1:** Data processing process of the convolutional neural network algorithm.

**Figure 2:** Data analysis process of the convolutional neural network topology analysis model based on big data and artificial intelligence strategies.

**Figure 3:** Simulation results of different tourism projects without big data coupling factors.

**Figure 4:** The simulation results of the dynamic coupling quantity value under the first-level big data coupling factor for the intelligent management types of different tourism projects.

**Figure 5:** The simulation results of the dynamic characterization of the two-level big data coupling factor for the intelligent management types of different tourism projects.

**Figure 6:** The simulation results of the dynamic characterization of the three-level big data coupling factor for the intelligent management types of different tourism projects.

**Figure 7:** Stability changes of management efficiency under different topological structures.

**Figure 8:** The results of topological analysis and verification on the management data of 3 types of different tourism projects.

**Figure 9:** Analysis of the accuracy of the data in the experimental results.

## Data Availability

The data used to support the findings of this study are available from the corresponding author upon request.
